RETRACTED

# MicroRNA-137 Upregulation Increases Bladder Cancer Cell Proliferation and Invasion by Targeting PAQR3

**DOI:** 10.1371/journal.pone.0109734

**Published:** 2014-10-16

**Authors:** Youcheng Xiu, Zan Liu, Shunyao Xia, Chengjun Jin, Huaifu Yin, Weiming Zhao, Qiong Wu

**Affiliations:** 1 School of Life Science and Biotechnology, State Key Laboratory of Urban Water Resource and Environment, Harbin Institute of Technology, Harbin, China; 2 Department of Urology, The First Affiliated Hospital of Harbin Medical University, Harbin, China; University of Barcelona, Spain

## Abstract

There is increasing evidence suggesting that dysregulation of some microRNAs (miRNAs) may contribute to tumor progression and metastasis and have been proposed to be key regulators of diverse biological processes such as transcriptional regulation, cell growth and tumorigenesis. Previous studies have shown that miR-137 is dysregulated in some malignancies, but its role in bladder cancer is still unknown. In our study, we find that miR-137 is up-regulated in human bladder cancer tissues and cell lines. Moreover, the higher level of miR-137 was associated with pM or pTNM stage in clinical bladder cancer patients. Enforced expression of miR-137 in bladder cancer cells significantly enhanced their proliferation, migration and invasion. Bioinformatics analysis identified the tumor suppressor gene PAQR3 as a potential miR-137 target gene. Further studies indicated that miR-137 suppressed the expression of PAQR3 by binding to its 3′-untranslated region. Silencing of PAQR3 by small interfering RNAs phenocopied the effects of miR-137 overexpression, whereas restoration of PAQR3 in bladder cancer cells bladder cancer cells overexpressing miR-137, partially reversed the suppressive effects of miR-137. These findings indicate that miR-137 could be a potential oncogene in bladder cancer.

## Introduction

Bladder cancer is the fifth most common cancer in the general population and the second most common cause of death in patients with genitourinary tract malignancies [1], [2]. More than 90% of urinary bladder tumors are comprised of transitional cell carcinoma (TCC) that arises from transitional epithelium [3]. Bladder tumors can be classified into two distinct categories: non-muscle and muscle invasive bladder cancer [4], [5]. Most bladder tumors (75–80%) are diagnosed as non-muscle-invasive tumors of which recurrence rates are high (50–70%) [6]. The rest are high-grade muscle invasive tumors (15%) that can rapidly progress to metastasis and lead to death [7]. Although considerable advances in treatment have been made, including improved surgical operation, radiotherapy and chemotherapy, bladder cancer continues to be a common disease with a high mortality rate [8], [9].

RETRACTED

Recently, increasing evidences suggest that a new class of RNAs, known as microRNAs (miRNAs), could regulate various target genes, including oncogenes and tumor suppressor [10]. miRNAs are endogenous 19∼22 nucleotide (nt) non-coding RNAs that can negatively regulate protein expression by inducing degradation of target mRNAs, impairing their translation or both by specifically binding to the 3′untranslated regions (3′UTR) of target mRNAs [11], [12]. An increasing number of studies have demonstrated that miRNAs contribute to most, if not all, basic biological processes, such as development, differentiation, apoptosis and cell proliferation [13]–[16]. Mutations of miRNA genes or dysregulation expression of miRNAs have been well described in many types of tumors, including gastric cancer, lymphoma, breast, lung, colon and liver cancers [17]–[22]. However, the role of miRNAs in bladder cancer remains largely unknown.

MiR-137 has attracted much attention because it is frequently down-regulated and functions as a tumor suppressor in many cancers such as ovarian cancer, gastric cancer, glioblastoma, lung cancer, colorectal cancer and neuroblastoma [23]–[28]. A previous study by Shimuzu et al. also showed that miR-137 was frequently methylated in primary bladder tumors and ectopic expression of miR-137 suppressed bladder cancer cell proliferation [29]. However, we herein report the contradictory expression and function of miR-137 in bladder cancer, which are opposed to that reported in the literature. In this study, we detected frequent upregulation of miR-137 in human bladder cancer tissues and cell lines. Overexpression of miR-137 promoted cell proliferation, migration and invasion of bladder cancer cells. Moreover, we found that PAQR3, a novel tumor suppressor gene, was the direct target of miR-137 in bladder cancer. Thus, our results suggest important roles for miR-137 in bladder cancer pathogenesis and indicate its potential application in cancer therapy.

## Materials and Methods

### Ethics statement

All of these patients agreed to participate in the study and gave written informed consent. Both this study and consent were approved by the ethical board of the institute of The First Affiliated Hospital of Harbin Medical University and complied with the Declaration of Helsinki.

### Human tissues

Biopsies from bladder cancer and the adjacent normal urothelium were obtained from patients undergoing radical cystectomy for bladder cancer at The First Affiliated Hospital of Harbin Medical University, China. The surgeries occurred from April 2010 to April 2013, and all patients provided signed informed consent. The biopsies were stored in liquid nitrogen immediately after resection until RNA extraction. The demographic and clinical pathologic data are listed in table S1.

RETRACTED

### Cell lines, cell culture and miRNA transfection

Four human bladder cancer cell lines T24, J82, 5637 and UMUC3 and one normal bladder cell line, SV-HUC-1, were purchased from the Shanghai Institute of Biochemistry and Cell Biology at the Chinese Academy of Sciences [30]. The cell lines were cultured in RPMI 1640 medium supplemented with 10% heat-inactivated fetal bovine serum under a humidified atmosphere of 5% CO2 at 37°C. The day before transfection, the cells were plated in growth medium without antibiotics at a density of 30–40%. The transfection of hsa-miR-137 mimic, inhibitor, and scramble, chemically synthesized by GenePharma (Shanghai, China) was performed using Lipofectamine 2000 (Invitrogen, Carlsbad, CA) according to the manufacturer’s protocol and were transfected into the cells with a final oligonucleotide concentration of 20 nmol/L.

### RNA isolation and qRT-PCR

Total RNA from tissue samples and cultured cells was isolated using TRIzol reagent (Takara, Dalian, China). Before performing Quantitative RT-PCR assays (qPCR), RNA was reverse-transcribed into miRNA cDNA and total cDNA using One Step PrimeScript miRNA cDNA Synthesis Kit (Takara, Dalian, China) and PrimeScript RT reagent Kit (Takara, Dalian, China), respectively. Real-time PCR primer sequences and conditions were listed in Table S2 and Table S3, respectively, according to the MIQE guideline. The mRNA and miRNA expression levels were detected by qPCR with Applied Biosystems 7500 Fast Real-Time PCR System real-time PCR System (Applied Biosystems, Carlsbad, USA) with SYBR Premix Ex Taq (Takara, Dalian, China) according to the manufacturer’s instructions and were normalized versus GAPDH mRNA and small nuclear RNA U6, respectively. The Ct value of miR-137 and PAQR3 was quantified with the 2^−ΔΔCt^ method.

### Migration and invasion assays

Cell invasion and migration were assayed using a transwell chamber (Millipore, USA) with and without Matrigel (BD, Franklin Lakes, USA). For the invasion assay, a transwell chamber was placed into a 24-well plate and was coated with 30 µl Matrigel and was incubated for forty minutes at 37°C. In both transwell assay, cells, 48 hours after transfected, were trypsinized and seeded in chambers at the density of 8×10^4^ cells per well and cultured in medium with RPMI 1640 medium with 2% serum, while 600 µl of 10% FBS-1640 was added to the lower chamber. Twentyfour hour’s later, migrated cells were fixed with 100% methanol for 30 min. Non-migrated Cells were removed by cotton swabs. Then cells on bottom surface of the membrane were stained by 0.1% crystal violet (Sigma) for 20 min. Cell images were obtained under a phase-contrast microscope (Olympus, Tokyo, Japan).

RETRACTED

### Cell proliferation

Cell proliferation assays were performed using a Cell Counting Kit-8 (Dojindo, Kumamoto, Japan). Bladder cancer cells were plated in 24-well plates at 2×10^5^ cells per well. Cells were incubated in 10% CCK-8 (Dojindo; Kumamoto, Japan) that was diluted in normal culture medium at 37°C until the visual color conversion occurred. Proliferation rates were determined at 0, 24, 48 and 72 hours after transfection.

### Western blots

Equivalent quantities (30–50 µg) of protein were separated by 10% SDS polyacrylamide gels and transferred to polyvinylidene fluoride (PVDF) membranes. Membranes were blocked with 5% non-fat dried milk and incubated overnight with the appropriate primary antibody at dilutions specified by the manufacturer. Next, the membranes were washed three times in TBST and incubated with the corresponding horseradish peroxidase (HRP)-conjugated secondary antibody at 1∶5,0000 dilution for 1 h. Bound secondary antibody was detected using the Enhanced Chemiluminescence (ECL) system (Pierce Biotechnology Inc, USA). Primary immunoblotting antibodies were: anti-GAPDH, anti-PAQR3 (Santa Cruz Biotechnology, USA).

### Luciferase assay

T24 cells were seeded in 24-well plates (1×10^5^ cells/well) and incubated for 24 h before transfection. For the reporter gene assay, the cells were cotransfected with 0.5 µg of pGL3-PAQR3-3′UTR or pGL3- PAQR3-3′UTR Mut plasmid, 0.05 ng of the phRL-SV40 control vector (Promega, USA), and 100 nM miR-137 or control RNA using Lipofectamine 2000 (Invitrogen, USA). The firefly and renilla luciferase activities were measured consecutively through a dual luciferase assay (Promega, USA) 24 h after transfection.

### Statistical analysis

Each experiment was repeated at least three times. Statistical analyses were performed using SPSS 15.0. Data are presented as the mean ± standard deviation. Statistical analyses were performed with either an analysis of variance (ANOVA) or Student’s t-test, and the statistical significance level was set at α = 0.05 (two-side).

## Results

### Expression of miR-137 is up-regulated in bladder cancer cell lines

The expression of miR-137 was first evaluated by quantitative reverse transcription-PCR (qRT-PCR) in bladder cancer cell lines and one normal bladder cell line SV-HUC-1. As shown in Fig. 1, miR-137 was significantly up-regulated in all the bladder cancer cell lines compared with SV-HUC-1. We further quantified the expression level of miR-137 in 6 pairs of human bladder cancer tissues and adjacent normal mucosal tissues by qRT-PCR (Fig. 1). The results showed that the expression level of miR-137 was generally higher in tumor tissues compared to matched non-tumor tissues. Thus, we speculated that miR-137 might be a putative oncogene in bladder cancer.

RETRACTED

**Figure 1:** The expression of miR-137 is up-regulated in bladder cancer cell lines. (A). Upregulation of miR-137 expression in bladder cancer cell lines and tissues compared with the corresponding controls. Relative expression of miR-137 in four bladder cancer cell lines and one normal bladder cell line SV-HUC-1 was determined by qRT-PCR. U6 snRNA was used as internal control. (B) Relative expression of miR-137 in 6 surgical specimens of bladder cancer tissues and matched non-tumor tissues was determined by qRTPCR. U6 snRNA was used as internal control.

### Expression of miR-137 in clinical bladder cancer patients and their correlation analysis with clinicopathological characteristics

To study the relationship of miR-137 with bladder cancer occurrence, the expression of miR-137 was detected in 50 clinical patients using real-time PCR. Out of 50 bladder cancer samples, miR-137 was up-regulated in 45 cases (45/50, 90%) compared with adjacent tissues (Fig. 2B). Meanwhile, miR-137 was down-regulated in 5 cases (5/50, 10%). In general, the expression of miR-137 in bladder cancer tissues was significant higher than in adjacent tissues (Fig. 2A, p<0.001). The higher level expression of miR-137 was associated with pTNM stage (Fig. 2C), and higher level of miR-137 was associated with pM stage (p = <0.05, metastasis vs. no metastssis) in bladder cancer patients (Fig. 2D). These data suggested that alterations of miR-137 could be involved in bladder cancer progression.

**Figure 2:** The expression of miR-137 in clinical bladder cancer patients and their correlation analysis with clinicopathological characteristics. (A) Relative miR-137 expression levels in bladder cancer tissues and adjacent normal tissues were determined by qRT-PCR. U6 snRNA was used as internal control. (B) miR-137 was detected in 50 pairs of bladder cancer tissues and its adjacent normal controls by quantitative RT-PCR. Data are presented as log2 of fold change of bladder cancer tissues relative to adjacent normal regions; (C) and (D) The Statistical analysis of the association between miRNA level and pTNM stage (I, II, III and IV) and pM stage (No metastasis and Metastasis); *p<0.05, and **p<0.01, ***p<0.001.

### Overexpression of miR-137 promoted bladder cancer cell proliferation, migration and invasion

We explored the potential impact of miR-137 in bladder cancer cell proliferation, migration and invasion. Cells were transfected with scrambled control oligo or miR-137 mimics and inhibitor, which showed high transfection efficiency (Fig. 3A). CCK-8 proliferation assay showed that cell proliferation was promoted in miR-137 mimics-transfected bladder cancer cells compared with scrambled oligo-transfected cells or untreated cells (Fig. 3B). Conversely, miR-137 inhibitor significantly inhibited the proliferation of the T24 cells (Fig. 3C). Intriguingly, migration and invasion assay showed that overexpression of miR-137 significantly promoted the migration and invasion of T24 cells compared with the control whereas miR-137 inhibitor inhibited both cell migration and invasion (Fig. 3D and E).

RETRACTED

**Figure 3:** Overexpression of miR-137 promoted bladder cancer cell proliferation, migration and invasion. (A) Expression levels of miR-137 were examined by real-time PCR after transfection of miR-137 mimics or sramble or no transfection. (B) Growth of T24 cells was shown after transfection with miR-137 mimics or sramble or no transfection. The growth index as assessed at 0, 24, 48 and 72 h. (C) Expression levels of miR-137 were examined by real-time PCR after transfection of miR-137 inhibitor or control or no transfection. (D) Growth of T24 cells was shown after transfection with miR-137 inhibitor or control or no transfection. The growth index as assessed at 0, 24, 48 and 72 h. (E) Transwell analysis of T24 cells after treatment with miR-137 mimics, inhibitors or scramble or control; the relative ratio of migrated cells per field is shown below. (D) Transwell analysis of T24 cells after treatment with miR-137 mimics, inhibitors or scramble or control; the relative ratio of invasive cells per field is shown below, *p<0.05, **p<0.01, and ***p<0.001.

### MiR-137 targets PAQR3 in bladder cancer cells

As predicted by PicTar, there was complementarity between has-miR-137 and the PAQR3 3′UTR (Fig. 4A). Overexpression of miR-137 reduced the protein and mRNA levels of PAQR3 in bladder cancer cells (Fig. 4C and D). The effect of miR-137 on the translation of PAQR3 mRNA into protein was then assessed by using a luciferase reporter assay (Fig. 4B). Enforced expression of miR-137 remarkably reduced the luciferase activity of the reporter gene with the wild-type construct but not with the mutant PAQR3 3′UTR construct, which indicates that miR-137 directly targeted the PAQR3 3′UTR.

**Figure 4:** miR-137 targets PAQR3 in bladder cancer cells. (A) Schematic representation of PAQR3 3′ UTRs showing putative miRNA target site. (B) The analysis of the relative luciferase activities of PAQR3-WT, PAQR3-MUT in T24 cells. The error bars are derived from triplicate expriments. (C) qRT-PCR analysis of PAQR3 mRNA expression in T24 cells after treatment with miR-137 mimics or scramble or no transfection. The expression of PAQR3 was normalized to GAPDH. (D) Western blot analysis of PAQR3 expression in T24 cells transfected with miR-137 mimics or scramble or no transfection. GAPDH was also detected as a loading control.

RETRACTED

### Restored expression of PAQR3 partially rescued miR-137-enhanced cell proliferation and invasion

We first analyzed the function of PAQR3 in bladder cancer cells. As shown in Fig. 5A, transfection of small interfering RNA against PAQR3 into T24 cells led to dramatically decreased PAQR3 protein expression. Silencing of PAQR3 significantly enhanced the proliferation of bladder cancer cells (Figs. 5B), which phenocopied the effects of miR-137 on proliferation of bladder cancer cells. Co-transfection of a construct expressing PAQR3 and miR-137 in T24 cells led to the restoration of PAQR3 expression, as confirmed by Western blot (Fig. 5C). This restoration of PAQR3 significantly inhibited the proliferation and invasive capabilities of bladder cancer cells. More importantly, we found that restoration of PAQR3 could significantly reverse the proliferation and invasion promoted by miR-137 (Figs. 5D and 5E). In summary, these data indicate that inhibition of PAQR3 expression by miR-137 is responsible, at least in part, for the promoting effects of miR-137 on cell proliferation and invasion in human bladder cancer.

**Figure 5:** The expression of PAQR3 partially rescued miR-137-enhanced cell proliferation and invasion. (A) Western blot analysis showed that transfection of small interfering RNA against PAQR3 into T24 cells led to dramatically decreased PAQR3 protein expression. GAPDH was also detected as a loading control. (B) Silencing of PAQR3 significantly enhanced the proliferation of bladder cancer cells. The growth index as assessed at 0, 24, 48 and 72 h. (C) Western blot analysis of PAQR3 in T24 cells co-transfected with either miR-137 mimic or scramble and 2.0 µg pCDNA- PAQR3 or pCDNA empty vector. GAPDH was also detected as a loading control. (D) Cell growth curves in T24 cells transfected with different combinations at 0, 24, 48 and 72 h. (E) Transwell analysis of T24 cells treated with different combinations. The relative ratio of invasive cells per field is shown right. *p<0.05, **p<0.01, ***p<0.001.

## Discussion

During the last decades, miRNAs have emerged as major regulators involved in diverse biological processes such as transcriptional regulation, cell differentiation and tumorigenesis [31]. Globally aberrant miRNA expression profiles of tumors have provided valuable insights into the molecular pathways of oncogenesis [32]. As one of the most prominent miRNAs implicated in the tumorigenesis, miR-137 has presented with a controversial role during tumor progression [33]. MiR-137 was found to be reduced in numerous human cancers, including gastric cancer, glioblastoma and breast cancer [24], [25], [34]. The exact role of miR-137 in bladder cancer was still unclear although its tumor-suppressing function has been implicated [29]. Thus, our current study intended to clarify the expression and biological function of miR-137 in bladder cancer. Contrary to the findings of Shimuzu et al. [29], our study demonstrated that miR-137 was frequently up-regulated in bladder cancer cell lines and tissues compared to normal bladder cell line and tissues. Based on these findings, we hypothesized that miR-137 might be a potential oncogene in bladder cancer. As expected, enforced expression of miR-137 enhanced proliferation, migration and invasion of T24 cells. The reasons of discrepancies between findings of the present study and that of Shimuzu et al. remain unclear but the ethnic background of clinical samples may play a role. Moreover, the oncogenic function of miR-137 may be specific to bladder tissue since its tumor suppressing function has been widely reported in other tissue types. Our present findings suggest that miR-137 plays a critical role in the invasive and metastatic potential of bladder cancer and may be potential diagnostic and predictive biomarkers.

RETRACTED

Next, we addressed the molecular mechanism of miR-137 in promoting proliferation, migration and invasion in bladder cancer cells. In this study, the real-time PCR, Western blots and luciferase assays showed that PAQR3 is a target of miR-137. Importantly, specific PAQR3 knockdown with siRNA phenocopied the migration- and invasion-promoting effects of miR-137 over-expression. We also showed that, when miR-137-expressing cells resumed PAQR3 expression, their invasion deficiencies were partly reversed. Therefore, we believe that miR-137 plays a role in the promotion of metastasis in bladder cancers, at least in part, by downregulating the protein expression of PAQR3. PAQR3 belongs to the progesterone and AdipoQ receptor (PAQR) family and is a seven-transmembrane protein specifically located at the Golgi apparatus in mammalian cells [35]. Previous studies have showed that PAQR3, also known as RKTG (Raf kinase trapping to Golgi), could act as a spatial regulator of Raf kinase by sequestering Raf to the Golgi apparatus [36]. PAQR3 functions as a tumor suppressor due to its inhibitory activity on Raf/MEK/ERK signaling [37]. When overexpressed in human A375 melanoma cells, a human malignant melanoma cell line with B-Raf mutation, PAQR3/RKTG inhibits ERK activation, cell proliferation and transformation of the cells [37]. Moreover, deletion of PAQR3 in mice led to increased incidence of skin tumorigenesis. PAQR3/RKTG also could inhibit cell proliferation, migration, sprouting and angiogenesis of endothelial cells, and the expression level of PAQR3 is significantly downregulated in clinical clear-cell renal cell carcinoma samples, with an inverse correlation with VEGF expression level [38]. Furthermore, previous studies have also indicated that PAQR3 has a functional interaction with p53 in cancer formation and epithelial-to-mesenchymal transition [39]. The expression level of PAQR3 was significantly decreased in colorectal cancer samples in comparison with adjacent normal tissues and the expression level of PAQR3 was inversely associated with tumor grade in the colorectal cancer samples [40]. Our studies also have showed that overexpression of PAQR3 can inhibit cell proliferation and invasion. Upregulation of these miRNAs in cancer may facilitate the expression of PAQR3, leading to enhanced metastasis of the cancer.

RETRACTED

In conclusion, our results have shown that miR-137 was significantly upregulated in bladder cancer cells and tissues. Enforced expression of miR-137 promoted bladder cancer cell proliferation, migration and invasion through directly targeting PAQR3. This novel miR-137/PAQR3 axis may provide new insights into the mechanisms underlying tumor metastasis, and repression of miR-137 expression may be a potential therapeutic strategy for the treatment of bladder cancer in the future.

## Supporting Information

Table S1 **Clinicopathologic charateristics of patients with bladder cancer.**
(DOCX)

Table S2 **Primer sequences.**
(DOC)

Table S3 **Checklist of MIQE guideline.**
(DOC)
